The article "Pest susceptibility, yield and fiber traits of transgenic cotton cultivars in Multan, Pakistan" was retracted in 2022. Reasons: compromised peer review; a conflict of interest; concerns about the authorship.

# Pest susceptibility, yield and fiber traits of transgenic cotton cultivars in Multan, Pakistan

**DOI:** 10.1371/journal.pone.0236340

**Published:** 2020-07-21

**Authors:** Haider Karar, Muhammad Amjad Bashir, Muneeba Haider, Najeeba Haider, Khalid Ali Khan, Hamed A. Ghramh, Mohammad Javed Ansari, Çetin Mutlu, Suilman Mohammad Alghanem

**Affiliations:** 1 Mango Research Institute, Multan, Pakistan; 2 Department of Plant Protection faculty of Agricultural Sciences, Ghazi University Dera Ghazi Khan Punjab, Dera Ghazi Khan, Pakistan; 3 Muhammad Nawaz Shareef University of Agriculture, Multan, Pakistan; 4 Research Center for Advanced Materials Science (RCAMS), King Khalid University, Abha, Saudi Arabia; 5 Unit of Bee Research and Honey Production, Faculty of Science, King Khalid University, Abha, Saudi Arabia; 6 Biology Department, Faculty of Science, King Khalid University, Abha, Saudi Arabia; 7 Department of Botany, Hindu College Moradabad, Moradabad, Uttar Pradesh, India; 8 Department of Plant Protection, Harran University, Şanlıurfa, Turkey; Bahauddin Zakariya University, PAKISTAN

## Abstract

Cotton (*Gossypium hirsutum* L.), being a cash and fiber crop is of high significance in Pakistan. Numerous insect pests and viral diseases in Pakistan and around the world attack cotton crop. Genetically modified cotton (transgenic, resistant to lepidopteran insects), hereafter written as ‘*Bt*-cotton’ has been introduced in many regions of the world to combat bollworms. However, cultivars differ in their pest susceptibility, yield response and fiber quality traits. Nonetheless, recent studies have indicated that lepidopteran pests are evolving resistance against ‘*Bt*-cotton’. Several ‘*Bt*-cotton’ cultivars have been developed in Pakistan in the past decade; however, limited is known about their pest susceptibility, seed-cotton yield and fiber quality traits. This two-year field study evaluated pest susceptibility, yield and fiber quality traits of thirteen newly developed ‘*Bt*-cotton’ cultivars in Pakistan. The cultivars differed in their susceptibility to sucking insects during both years of study. The cultivars ‘FH-647’, ‘SLH-8’, ‘FH-Lalazar’ and ‘IUB-013’ were more susceptible to jassid, whereas ‘BS-52’ exhibited higher susceptibility to whitefly during both years of study. Similarly, cultivars ‘AGC-999’ and ‘MNH-992’ proved highly susceptible to thrips during each study year. Although ‘*Bt-*cotton’ is resistant to bollworms, cultivars ‘SLAH-8’, ‘VH-305’ and ‘BH-184’ were susceptible to spotted bollworm, while ‘SLAH-8’, ‘RH-647’ and ‘VH-305’ were infested by American bollworm. The most susceptible cultivars to cotton leaf curl virus (CLCuV) attack were ‘RH-647’, ‘IR-NIBGE-7’ and ‘VH-305’. The highest seed-cotton yield was recorded for ‘FH-Lalazar’ during both years of study. Similarly, the highest ginning out turn was recorded for cultivars ‘BS-52’, ‘VH-305’, ‘RH-647’, ‘IUB’ and ‘AA-919’. The cultivar ‘FH-Lalazar’ exhibited low pest susceptibility and CLCuV infestation compared to the rest of cultivars. The highest and the lowest gross and net incomes and benefit:cost ratio were noted for ‘FH-Lalazar’ and ‘RH-647, respectively. Keeping in view the low pest susceptibility and high seed-cotton yield, ‘FH-Lalazar’ could be recommended for higher yield and economic returns in Multan, Pakistan. Nonetheless, regional trials should be conducted for site-specific or region-specific recommendations.

The article "Pest susceptibility, yield and fiber traits of transgenic cotton cultivars in Multan, Pakistan" was retracted in 2022. Reasons: compromised peer review; a conflict of interest; concerns about the authorship.

## Introduction

Cotton (*Gossypium hirsutum* L.), being an oilseed and fiber crop is considered as backbone of Pakistan’s national economy [1, 2]. Cotton contributes 7.8% towards value addition in agriculture and fulfils 55% of country’s domestic cooking oil requirements [3]. Numerous insect pests and diseases attack cotton crop, which reduce seed-cotton yield and hamper fiber quality [4]. Globally, 1326 insect species have been reported on cotton [5], of which 10–15 incur monetary losses [6]. These species are major constraint in cotton production [6]. The management of different cotton pests has been a challenging task for agricultural experts and cotton growers. It is estimated that insect infestation causes ~20–40% annual yield and quality losses of cotton in Pakistan [7, 8].

The introduction of ‘*Bt*-cotton’ (genetically modified, transgenic, and insect-resistant) in Pakistan was a major relief to farmers for lowering the damages caused by bollworms. The ‘*Bt*-cotton’ is resistant to bollworms; however, provides no control of sucking pests. The risk of bollworms’ damage, especially of *Heliothis armigera* reduced after the introduction of ‘*Bt*-cotton’; however, the problem of pink bollworm still persists [9]. Several recent studies have indicated that ‘*Bt*-cotton’ is loosing resistance against bollworms [10–12]. Furthermore, pink bollworm have sustained resistance against ‘*Bt*-cotton’ [13, 14]. Cotton pest management in Pakistan relies on excessive use of insecticides. Insecticides play a key role in pest management; however, their non-judicious use negatively affects the sustainability of agro-ecosystems [15]. On the other hand, insecticides pose adverse effects to environment, natural enemies and human health. Nonetheless, recent study by Shahzad et al. [16] have indicated that cotton yield and nitrogen use efficiency is low in Pakistan compared to developed world.

Constant use of insecticides has necessitated the adoption of integrated pest management (IPM) approaches in cotton and other crops in the country. The IPM is very useful in lowering the losses caused by pests; thus, enhances the sustainability of agro-ecosystems [17]. A sustainable IPM approach could lower the reliance of farming community on insecticides. Inducing host plant resistance (HPR) is a globally-known strategy in wake of IPM. This mechanism is used globally to save economically important plants from pest attack, which increases their yield [18]. The HPR is compatible, cost-effective and ecologically safe than rest of the pest control tactics [19–22]. The use of ‘*Bt*-cotton’ is induction of HPR for IPM of cotton pests [23]. The use of resistant cultivars lay a strong foundation of IMP program, and provide excellent pest management when combined with other pest control methods. Insect-resistant transgenic crops could be an important IPM tool because of their potential to lower insecticide use [24, 25]. However, exploring the resistance level to pests and yield of different cultivars is a pre-requisite for their use in IMP programs. Several ‘*Bt*-cotton’ cultivars have been developed in Pakistan in last decade; however, nothing is known about their pest susceptibility and yield response under field conditions.

The article "Pest susceptibility, yield and fiber traits of transgenic cotton cultivars in Multan, Pakistan" was retracted in 2022. Reasons: compromised peer review; a conflict of interest; concerns about the authorship.

This two-year field study investigated the pest susceptibility, seed-cotton yield and fiber quality traits of thirteen newly-developed ‘*Bt*-cotton’ cultivars in Multan, Pakistan.

## Materials and methods

### Experimental site and cultivars

The current study was conducted at Cotton Research Station, Multan, Pakistan during cotton growing seasons of 2014 and 2015. Thirteen newly developed ‘*Bt*-cotton’ cultivars developed/marketed by different public and private institutes in Pakistan were used in the study. The details regarding names, developing institute and their nature (i.e., public or private) are presented in Table 1.

**Table 1:** List of different transgenic cotton cultivars used in the study and their manufacturers.

Cultivars	Institute/Developer	City	Institute type
**AGC-999**	Allah Din group of Companies	Multan	Private
**BS-52**	Bandaisha Seed	Multan	Private
**CYTO-177**	Central Cotton Research Institute	Multan	Government
**RH-647**	Cotton Research Station	Rahim Yar Khan	Government
**IUB-013**	Islamia University	Bahawalpur	Government
**AA-919**	Ali Akbar Group	Multan	Private
**SLH-8**	Cotton Research Station	Sahiwal	Government
**BH-184**	Regional Research Institute	Bahawalpur	Government
**FH-Lalazar**	Cotton Research Institute	Faisalabad	Government
**VH-305**	Cotton Research Station	Vehari	Government
**MNH-992**	Cotton Research Station	Multan	Government
**NIAB-878B**	Nuclear Institute for Agriculture and Biology	Faisalabad	Government
**IR-NIBGE-7**	Nuclear Institute for Biology and Genetic Engineering	Faisalabad	Government

The seeds of all cultivars were purchased from respective institutes. The seeds were sown on finely prepared seedbed on May 27, 2014 and May 24, 2015 during 1^st^ and 2^nd^ year of the study. Soil samples were collected from the experimental site to assess the physiochemical properties before initiating the experiment each year. The samples were collected following the procedures opted in Onen et al. [26], whereas analyses were performed following the soil analyses procedures described by Farooq et al. [27]. The soil properties of the experimental site during both study years are summarized in Table 2.

The article "Pest susceptibility, yield and fiber traits of transgenic cotton cultivars in Multan, Pakistan" was retracted in 2022. Reasons: compromised peer review; a conflict of interest; concerns about the authorship.

**Table 2:** Physiochemical properties of experimental soil during both years of study.

	Unit	Year-I	Year-II
**Chemical properties**			
Organic matter content	%	0.48	0.57
Total nitrogen (N)	%	0.07	0.08
Available phosphorus (P)	mg kg^-1^	8.06	9.01
Available potassium (K)	mg kg^-1^	215.50	229.60
pH		8.37	8.49
EC	dS m^-1^	4.76	5.21
**Physical properties**			
Silt	%	49.25	55.10
Sand	%	29.60	25.40
Clay	%	21.15	19.50
Textural class		Silty-clay	Silty-clay

The experimental field was irrigated before seedbed preparation. The seedbed was prepared once the soil reached workable moisture regime, with two ploughings followed by planking. Seeds were sown with a manual drill by keeping row-to-row and plant-to-plant distance at 75 and 30 cm, respectively. Seed rate was kept 25 kg ha^-1^. The net plot size was 5 × 3 m and each treatment was replicated three times. The recommended field practices by Department of Agriculture Extension (http://www.agripunjab.gov.pk/) for the crop season were opted throughout the experiment. The weather data collected form the experimental site for both study years is given in Table 3.

**Table 3:** Weather data collected from the experimental site during both years of study.

Month	Temperature (ºC)	Relative humidity (%)	Sunshine (hours)	Total rainfall (mm)
**Year-I**				
May	35.3	72.6	8.9	12.0
June	36.4	67.2	9.3	14.0
July	34.0	71.1	8.1	26.8
August	32.6	81.3	7.3	111.0
September	30.7	80.2	7.1	13.0
October	26.0	65.4	6.9	0.0
November	18.6	64.3	3.8	0.0
December	15.6	76.4	3.2	0.0
**Year-II**				
May	33.2	60.9	9.8	20.1
June	34.8	72.1	8.5	35.7
July	33.6	71.2	8.2	34.2
August	30.8	81.6	7.1	113.7
September	29.4	74.3	7.0	14.0
October	27.0	72.2	6.4	0.0
November	17.4	79.4	3.9	4.2
December	15.2	77.5	3.6	0.0

The values are monthly averages for the respective month

### Population monitoring of sucking insects

Population of sucking insects such as jassid (either adults or nymphs), whitefly (adults) and thrips (either adults and nymphs) per leaf was monitored at weekly intervals starting from July, 24 to September, 18, 2014 during both years of study. The presence of adults or nymphs was monitored early in the morning. Fifteen randomly leaves selected from fifteen different plants were monitored and presence of the sucking insects was recorded. The random leaf selection sequence was; first leaf from upper one third of the first plant, second leaf from middle of the second plant and third leaf from the lower portion of the third plant. The average population/leaf was calculated by using Eq 1,

$$X=\frac{X_{1}+X_{2}+X_{3}\ldots \ldots \ldots ..{+X}_{n}}{N}$$ Eq 1

Here, N = total numbers of leaves observed, X = Mean number of adults + nymphs per leaf and X_1_+X_2_+X_3_+ ···· X_n_ = Number of insects observed per leave

The article "Pest susceptibility, yield and fiber traits of transgenic cotton cultivars in Multan, Pakistan" was retracted in 2022. Reasons: compromised peer review; a conflict of interest; concerns about the authorship.

### Population monitoring of bollworms

The larval population of spotted, American and pink bollworms was monitored from ten randomly plants. Furthermore, the number of rosette flowers were recorded at weekly interval. Average population of bollworms was calculated by Eq 1 described above. The larval population of pink bollworm in the left over bolls was recorded by plucking the total left over bolls from each plot and kept in lab for 3–4 days. Subsequently the bolls were opened with knife and pink bollworm larvae were counted. Percent damage due to larvae was calculated by Eq 2.

$$\mathrm{Damage}\;(\%)=\frac{\mathrm{Number}\;\mathrm{of}\;\mathrm{bolls}\;\mathrm{infested}\;\mathrm{with}\;\mathrm{pink}\;\mathrm{bollworm}}{\mathrm{Total}\;\mathrm{number}\;\mathrm{of}\;\mathrm{bolls}}\times 100$$ Eq 2

### Cotton leaf curl virus (CLCuV) incidence

The incidence of cotton leaf curl virus (CLCuV) was determined by counting all healthy and affected plants in each experimental unit at 30, 60, 90 and 120 days after sowing (DAS). The CLCuV incidence was calculated by using Eq 3:

$$\mathrm{CLCuV}\;\mathrm{incidence}\;(\%)=\frac{\mathrm{CLCuV}\;\mathrm{infested}\;\mathrm{plants}}{\mathrm{Total}\;\mathrm{numebr}\;\mathrm{of}\;\mathrm{plants}}\times 100$$ Eq 3

### Insecticide application

The populations of sucking insects and bollworms were monitored within economic threshold level (ETL). The pest population was kept below ETL to observe the actual seed-cotton yield. Therefore, crop was sprayed with appropriate insecticides at field recommended doses for respective insects once their population just crossed ETL.

### Seed-cotton yield

Total seed-cotton yield was recorded for each studied cultivar during each study year. The seed-cotton was manually picked at regular intervals once the bolls were open from all plants in each experimental unit. A total 6 pickings were done for all experimental units and seed-cotton yield of all pickings was added to get total yield. Then the seed-cotton yield was converted to per hectare by unitary method.

The article "Pest susceptibility, yield and fiber traits of transgenic cotton cultivars in Multan, Pakistan" was retracted in 2022. Reasons: compromised peer review; a conflict of interest; concerns about the authorship.

### Fiber characteristics and quality traits

The manually picked seed-cotton was dried under sun for three days. Afterwards, three random samples were taken from each seed-cotton lot of each cultivar. These samples were ginned by experimental small ginning machine. The ginning out turn percentage was calculated by Eq 4;

$$\mathrm{Ginning}\;\mathrm{out}\;\mathrm{turn}\;(\%)=\frac{\mathrm{Lint}\;\mathrm{weight}}{\mathrm{Seed}‐\mathrm{cotton}\;\mathrm{weight}}\times 100$$ Eq 4

Forty gram lint was taken from each sample and sent to fiber testing laboratory, Cotton Research Station, Multan for the fiber quality analysis. Staple length (mm), fiber fineness (μ g/inch) and fiber strength (g/tex) were analyzed. The fiber traits were measured on HVI spectrum^-1^ (Manufacturer Uster, USA).

### Statistical analysis

The difference between years were tested by two-way analysis of variance (ANOVA), which indicated significant difference for year × experiment interaction. Therefore, the data of both years were analyzed and represented separately. The collected data were subjected to Shapiro-Wilk normality test, which indicated a non-normal distribution. Therefore, data were normalized by Arcsine transformation technique to meet the normality assumption of ANOVA. One-way ANOVA was used to test the significance in the collected data. Tukey’s Honestly Significant Difference (HSD) test at 5% probability level was used to separate means where ANOVA indicated significant differences. The ANOVA was performed on Statistix software (version 8.1; Lawes Agricultural Trust Rothamsted Experimental Station, Rothamsted, UK). There was no CLCuV infestation at 30 DAS; therefore, it was excluded from the analysis and infestation data of 60, 90 and 120 DAS was included in the analysis.

### Economic analysis

An economic analysis was performed to assess the net benefits of the studied transgenic cotton cultivars. Total expenses incurred to raise the crop included the costs incurred on seed purchase, seedbed preparation, sowing, weed management, irrigation, fertilizing, harvesting and land rent for six months. Since there were no changes in the incurred cost, it remained similar for all of the cultivars. Gross income was estimated by using the existing price of seed-cotton in the local market. Net income was computed by subtracting the total expenses from gross income, and benefit:cost ratio (BCR) was recorded by dividing gross income with total production cost.

## Results

### Population of sucking insects

The tested cultivars significantly (Table 4) differed for their susceptibility to jassid population during both years of study. The highest jassid population was recorded on cultivar ‘RH-647’, during both years of study, which was statistically similar to cultivars ‘SLH-8’, ‘FH-Lalazar’ and ‘IUB-013’. The lowest jassid population was recorded on cultivars ‘VH-305’, ‘MNH-992’, ‘BH-184’ and ‘CYTO-177’ during both years of study (Table 5).

The article "Pest susceptibility, yield and fiber traits of transgenic cotton cultivars in Multan, Pakistan" was retracted in 2022. Reasons: compromised peer review; a conflict of interest; concerns about the authorship.

**Table 4:** Analysis of variance of pest infestation, yield and fiber quality traits of transgenic cotton cultivars.

Variable	SS	MS	F value	P value
**Jassid population**	1.91	0.16	198.14	< 0.0001*
**Whitefly population**	701.39	58.45	199.45	< 0.0001*
**Thrips population**	172.66	14.39	108.16	< 0.0001*
**Earis population**	21.11	1.76	57.83	< 0.0001*
**Heliothus population**	0.31	0.03	7.15	< 0.0001*
**Pink bollworm population**	3042.88	253.57	242.38	< 0.0001*
**CLCuV 60 DAS**	2472.26	206.02	84.58	< 0.0001*
**CLCuV 90 DAS**	9097.03	758.09	230.98	< 0.0001*
**CLCuV 120 DAS**	11430.26	952.52	271.16	< 0.0001*
**Seed-cotton yield**	11283089.60	940257.47	164.76	< 0.0001*
**Ginning out turn**	237.75	19.81	24.40	< 0.0001*
**Staple length**	76.26	6.36	8.00	< 0.0001*
**Fiber fineness**	22.97	1.91	49.51	< 0.0001*
**Fiber strength**	155.81	12.98	53.66	< 0.0001*
**Gross income**	4831308.07	402609.01	164.76	< 0.0001
**Net income**	4831308.07	402609.01	164.76	< 0.0001
**Benefit:cost ratio**	7.32	0.61	164.76	< 0.0001
**Year-II**				
**Jassid population**	1.83	0.15	203.29	< 0.0001*
**Whitefly population**	575.92	47.99	165.65	< 0.0001*
**Thrips population**	212.01	17.67	159.45	< 0.0001*
**Earis population**	27.23	2.27	67.72	< 0.0001*
**Heliothus population**	1.03	0.09	184.15	< 0.0001*
**Pink bollworm population**	2776.60	231.38	220.62	< 0.0001*
**CLCuV 60 DAS**	2782.25	231.85	10.59	< 0.0001*
**CLCuV 90 DAS**	9187.73	765.64	192.74	< 0.0001*
**CLCuV 120 DAS**	11528.41	960.70	238.65	< 0.0001*
**Seed-cotton yield**	12150692.23	1012557.69	175.54	< 0.0001*
**Ginning out turn**	223.43	18.62	32.35	< 0.0001*
**Staple length**	90.31	7.53	35.07	< 0.0001*
**Fiber fineness**	24.15	2.01	52.07	< 0.0001*
**Fiber strength**	166.15	13.85	33.19	< 0.0001*
**Gross income**	4784058.49	398671.54	175.54	< 0.0001
**Net income**	4784058.49	398671.54	175.54	< 0.0001
**Benefit:cost ratio**	7.32	0.61	175.54	< 0.0001

Source of variation = transgenic cotton cultivars, degree of freedom = 12, SS = sum of squares, MS = mean squares

* = significant (HSD ≤ 0.05), CLCuV = cotton leaf curl virus, DAS = days after sowing

**Table 5:** The infestation of different sucking insects and bollworms on transgenic cotton cultivars included in the study.

Population (numbers per plant of leaf)						
	Sucking insects			Bollworms		
Cultivars	Jassid	Whitefly	Thrips	Spotted	American	Pink
**Year-I**						
**BS-52**	0.68 d	15.84 a	5.09 b	0.00 d	0.00 b	44.47 i
**RH-647**	0.93 a	2.74 g	1.44 e	0.31 c	0.00 b	57.55 g
**FH-Lalazar**	0.88 b	7.31 d	0.95 efg	0.00 d	0.00 b	64.28 d
**VH-305**	0.40 f	2.41 g	2.53 d	1.05 b	0.00 b	60.04 e
**SLH-8**	0.93 a	2.86 fg	0.47 g	2.62 a	0.33 a	56.37 gh
**BH-184**	0.27 g	2.28 g	0.62 fg	0.86 b	0.00 b	77.26 b
**IR-NIBGE-7**	0.62 e	3.08 fg	2.56 d	0.00 d	0.00 b	58.09 fg
**MNH-992**	0.41 f	5.20 e	5.94 a	0.00 d	0.00 b	64.62 d
**CYTO-177**	0.27 g	10.32 c	1.14 ef	0.00 d	0.00 b	59.41 ef
**AGC-999**	0.60 e	12.72 b	6.41 a	0.00 d	0.00 b	79.13 a
**NIAB-878B**	0.68 d	5.97 e	4.31 c	0.00 d	0.00 b	60.07 e
**IUB-013**	0.80 c	2.86 fg	0.48 g	0.00 d	0.00 b	55.26 h
**AA-919**	0.72 d	3.69 f	0.66 fg	0.00 d	0.00 b	68.47 c
**HSD 0.05**	**0.047**	**0.908**	**0.61**	**0.29**	**0.1**	**1.71**
**Year-II**						
**BS-52**	0.59 d	14.58 a	5.52 b	0.00 e	0.16 b	45.62 h
**RH-647**	0.94 a	2.34 g	1.72 e	0.32 d	0.00 c	56.40 ef
**FH-Lalazar**	0.78 b	6.76 d	1.15 fg	0.00 e	0.00 c	63.06 c
**VH-305**	0.47 f	2.00 g	3.29 d	1.66 b	0.00 c	58.47 d
**SLH-8**	0.90 a	2.64 fg	0.85 g	2.71 a	0.60 a	54.90 fg
**BH-184**	0.34 g	1.87 g	1.01 fg	1.26 c	0.00 c	75.86 a
**IR-NIBGE-7**	0.52 e	2.76 fg	2.95 d	0.00 e	0.00 c	56.64 e
**MNH-992**	0.32 g	4.82 e	7.29 a	0.00 e	0.00 c	63.36 c
**CYTO-177**	0.23 h	9.11 c	1.43 ef	0.00 e	0.00 c	58.02 de
**AGC-999**	0.77 b	11.03 b	7.33 a	0.00 e	0.00 c	77.57 a
**NIAB-878B**	0.75 bc	5.15 e	4.87 c	0.00 e	0.00 c	58.94 d
**IUB-013**	0.71 c	2.52 g	1.09 fg	0.00 e	0.00 c	53.99 g
**AA-919**	0.63 d	3.46 f	1.05 fg	0.00 e	0.00 c	67.21 b
**HSD 0.05**	**0.046**	**0.89**	**0.55**	**0.3**	**0.03**	**1.73**

Means sharing same letter within a column are statistically non-significant (p > 0.05), HSD = honestly significant difference

Different cotton cultivars significantly differed for their susceptibility to whitefly during both years of study (Table 4). The highest whitefly population was recorded on cultivar ‘BS-52’ followed by ‘AGC-999’ and ‘CYTO-177’ during both years. The lowest whitefly population was observed on cultivars ‘VH-305’ ‘RH-647’ and ‘BH-184’ (Table 5).

The article "Pest susceptibility, yield and fiber traits of transgenic cotton cultivars in Multan, Pakistan" was retracted in 2022. Reasons: compromised peer review; a conflict of interest; concerns about the authorship.

Significant differences were observed among tested cultivars for thrips population during each study year (Table 4). The most dense thrips population was recorded on cultivar ‘AGC-999’, which was statistically at par with ‘MNH-992’. The lowest thrips infestation was recorded on ‘IUB-013’ and ‘SLH-8’ during 1^st^ and 2^nd^ year, respectively (Table 5).

### Population of bollworms

The tested cultivars significantly differed in supporting spotted bollworm population during both study years (Table 4). The highest number of spotted bollworms were recorded on cultivar ‘SLH-8’ during each study year, which was followed by ‘VH-305’ and ‘BH-184’ (Table 5).

American bollworm population ranged from 0.00 to 0.33 and 0.00–0.60 during 1^st^ and 2^nd^ year respectively. Similarly, no rosette flower was observed on any of the tested cultivars. Significant differences were noted among tested cultivars for pink bollworm population in left over bolls (Table 4). The highest number of pink bollworm larvae were recorded on cultivar ‘AGC-999’ and ‘BH-184’ during both years of study. The cultivar ‘BS-52’ had the lowest number of pink bollworms in left over bolls during both years of study (Table 5).

### Cotton leaf curl virus (CLCuV) incidence

No CLCuV infestation was recorded at 30 days after sowing (DAS) during both years of study. However, CLCuV incidence started to increase with the passage of time. Tested cultivars significantly differed for their susceptibility to CLCuV (Table 4). The highest CLCuV infestation at 60 DAS was recorded for cultivars ‘RH-647’, ‘MNH-992’ and ‘IR-NIBGE-7’, whereas the lowest infestation was recorded for ‘NIAB-878B’ during both years (Table 6). Similarly, the highest and the lowest CLCuV infestation 90 DAS was observed for cultivars ‘RH-647’and ‘VH-305’, and ‘MNH-992’, respectively (Table 6).

**Table 6:** Cotton leaf curl virus infestation on transgenic cotton cultivars included in the study.

	Year-I			Year-II		
Cultivars	CLCv60 (%)	CLCv90 (%)	CLCv120 (%)	CLCv60 (%)	CLCv90 (%)	CLCv120 (%)
**BS-52**	28.00 b	49.67 e	60.00 de	30.53 ab	53.85 e	62.50 cd
**RH-647**	29.00 ab	78.33 a	90.67 a	31.47 ab	82.33 a	93.17 a
**FH-Lalazar**	13.33 ef	46.00 f	58.00 ef	16.03 de	50.00 f	60.83 de
**VH-305**	28.67 ab	68.00 b	86.67 b	30.86 ab	70.83 b	90.83 a
**SLH-8**	10.33 g	56.00 d	63.00 d	13.53	59.83 d	65.50 c
**BH-184**	24.67 c	67.67 b	75.00 c	36.14 e	70.80 b	79.17 b
**IR-NIBGE-7**	30.00 ab	61.67 c	89.00 ab	32.25 a	66.00 c	92.83 a
**MNH-992**	31.00 a	34.33 gh	56.00 fg	33.11 ab	37.20 gh	58.17 ef
**CYTO-177**	19.00 d	33.00 hi	41.67 h	21.70 cd	36.37 h	45.17 g
**AGC-999**	11.00 fg	32.00 hi	40.00 h	13.50 e	36.15 h	44.17 g
**NIAB-878B**	9.67 g	37.00 g	57.33 ef	12.37 e	40.20 g	60.83 de
**IUB-013**	23.00 c	31.00 i	41.33 h	25.47 bc	34.27 h	44.83 g
**AA-919**	14.00 e	45.00 f	53.00 g	16.40 de	48.83 f	55.50 f
**HSD 0.05**	**2.61**	**3.04**	**3.14**	**7.85**	**3.34**	**3.36**

Means sharing same letter within a column are statistically non-significant (p > 0.05), CLCuV = cotton leaf curl virus, 60, 90 and 120 represent infestation at 60, 90 and 120 days after sowing, HSD = honestly significant difference

The highest infestation at 120 DAS was recorded for cultivars ‘RH-647’, ‘IR-NIBGE-7’ and ‘VH-305’. Likewise, the lowest infestation was recorded for cultivars ‘AGC-999’ and ‘IUB-013’ during both years (Table 6).

The article "Pest susceptibility, yield and fiber traits of transgenic cotton cultivars in Multan, Pakistan" was retracted in 2022. Reasons: compromised peer review; a conflict of interest; concerns about the authorship.

### Seed-cotton yield

Highly significant differences were recorded among tested cultivars for seed-cotton yield during both years (Table 4). The highest seed-cotton yield was recorded for cultivar ‘FH-Lalazar’ followed by cultivars ‘VH-305’, ‘AGC-999’, ‘MNH-992’, ‘CYTO-177’ and ‘BS-52’ during both years of study (Table 7). The lowest seed-cotton yield was recorded for cultivar ‘RH-647’ (Table 7).

**Table 7:** Yield and fiber quality traits of different transgenic cotton cultivars included in the study.

Cultivars	Seed-cotton yield (kg ha^-1^)	GOT (%)	Staple length (mm)	Fiber fineness (μg inch^-1^)	Fiber strength (g tex^-1^)
**Year-I**					
**BS-52**	2123 cd	46.98 bcd	27.17 a	5.83 bc	33.70 b
**RH-647**	1289 h	49.18 a	25.00 bc	5.78 cd	28.74 f
**FH-Lalazar**	3487 a	47.08 bc	26.03 ab	5.47 de	30.39 d
**VH-305**	2535 b	42.69 f	23.99 cd	5.25 ef	34.96 a
**SLH-8**	1905 e	48.06 ab	23.20 de	6.29 a	30.65 cd
**BH-184**	2008 de	42.52 f	25.43 bc	4.50 g	35.00 a
**IR-NIBGE-7**	1441 g	45.91 cde	24.60 bcd	4.94 f	31.40 c
**MNH-992**	2416 b	41.01 g	24.88 bc	5.40 e	30.40 d
**CYTO-177**	2169 c	47.26 bc	26.03 ab	6.14 ab	30.26 de
**AGC-999**	2477 b	42.18 fg	24.00 cd	5.19 ef	30.55 d
**NIAB-878B**	1981 e	45.05 e	27.33 a	3.35 h	29.49 ef
**IUB-013**	1934 e	43.33 f	25.23 bc	6.23 a	30.59 cd
**AA-919**	1631 f	45.55 de	22.27 e	5.32 e	29.00 f
**HSD 0.05**	**126.78**	**1.51**	**1.49**	**0.33**	**0.82**
**Year-II**					
**BS-52**	2169 e	47.82 cd	27.92 ab	6.26 bc	33.51 b
**RH-647**	1420 i	50.37 a	25.28 f	6.17 cd	29.91 f
**FH-Lalazar**	3698 a	48.32 bc	26.84 cd	5.92 de	32.03 cd
**VH-305**	2688 b	43.88 h	25.37 f	5.44 f	36.52 a
**SLH-8**	2004 f	49.45 ab	25.30 f	6.50 ab	32.33 cd
**BH-184**	2154 e	43.86 h	26.25 de	4.88 g	36.39 a
**IR-NIBGE-7**	1556 h	47.04 de	25.32 f	5.05 g	32.81 bc
**MNH-992**	2514 c	41.96 i	25.55 ef	5.69 ef	31.68 de
**CYTO-177**	2299 d	48.26 bcd	27.24 bc	6.45 abc	29.71 f
**AGC-999**	2619 bc	44.50 gh	26.04 ef	5.59 f	32.37 cd
**NIAB-878B**	2104 ef	46.15 ef	28.68 a	3.68 h	30.78 ef
**IUB-013**	2101 ef	44.61 gh	25.59 ef	6.67 a	31.84 cde
**AA-919**	1735 g	45.63 fg	22.17 g	5.44 f	30.36 f
**HSD 0.05**	**128.31**	**1.27**	**0.78**	**0.32**	**1.08**

Means sharing same letter within a column are statistically non-significant (p > 0.05), HSD = honestly significant difference

### Fiber quality traits

The tested cultivars significantly differed for fiber quality traits during both years (Table 4). The highest GOT was recorded for cultivar ‘RH-647’ during each year. The lowest GOT was recorded for ‘MNH-992’ (Table 7). The maximum staple length was recorded for cultivars ‘BS-52’ and ‘NIAB-878B’ during both years, which is a little below the standard 27.5 mm; however, was better as compared with rest of the cultivars. The minimum staple length was recorded for cultivar ‘AA-919’ (Table 7). Similarly, minimum fiber fineness was recorded for cultivar ‘SLH-8’ and ‘IUB-013’ during each year, whereas maximum fineness was recorded for cultivars ‘NIAB-878B’ (Table 7). The maximum fiber strength (35.0) was recorded for cultivars ‘BH-184’ and ‘VH-305’ as compared with standard fiber strength i.e., 30±2, whereas minimum was recorded for cultivars ‘RH-647’ and ‘AA-919’ cultivars during each study year (Table 7).

The article "Pest susceptibility, yield and fiber traits of transgenic cotton cultivars in Multan, Pakistan" was retracted in 2022. Reasons: compromised peer review; a conflict of interest; concerns about the authorship.

### Economic analysis

Gross and net incomes, and benefit:cost ratio (BCR) were significantly altered by different cultivars included in the study (Table 4). The production cost did not differ among cultivars due to similar cultural practices. The highest gross and net incomes and BCR were recorded for ‘FH-Lalazar’, whereas the lowest values of these were noted for ‘RH-647’ during both years of study (Table 8).

**Table 8:** Economic analysis of different transgenic cultivars grown under agro-climatic conditions of Multan, Pakistan.

Cultivars	Total expenditures US$ ha^-1^	Gross income US$ ha^-1^	Net income US$ ha^-1^	BCR
	Year-1			
**FH-Lalazar**	812.68	2282.24 a	1469.55 a	2.81 a
**VH-305**	812.68	1658.82 b	846.13 b	2.04 b
**AGC-999**	812.68	1621.20 b	808.51 b	1.99 b
**MNH-992**	812.68	1581.36 b	768.67 b	1.95 b
**CYTO-177**	812.68	1419.83 c	607.14 c	1.75 c
**BS-52**	812.68	1389.80 cd	577.12 cd	1.71 cd
**BH-184**	812.68	1314.32 de	501.64 de	1.62 de
**NIAB-878B**	812.68	1296.84 e	484.15 e	1.60 e
**IUB-013**	812.68	1265.60 e	452.91 e	1.56 e
**SLH-8**	812.68	1246.91 e	434.23 e	1.53 e
**AA-919**	812.68	1067.35 f	254.67 f	1.31 f
**IR-NIBGE-7**	812.68	943.12 g	130.43 g	1.16 g
**RH-647**	812.68	843.69 h	31.01 h	1.04 h
**HSD 0.05**	-	**82.96**	**82.96**	**0.10**
	**Year-II**			
**FH-Lalazar**	808.26	2320.84 a	1512.58 a	2.87 a
**VH-305**	808.26	1686.66 b	878.40 b	2.09 b
**AGC-999**	808.26	1643.37 bc	835.11 bc	2.03 bc
**MNH-992**	808.26	1577.87 c	769.61 c	1.95 c
**CYTO-177**	808.26	1442.65 d	634.40 d	1.78 d
**BS-52**	808.26	1361.41 e	553.16 e	1.68 e
**BH-184**	808.26	1352.14 e	543.88 e	1.67 e
**NIAB-878B**	808.26	1320.65 ef	512.40 ef	1.63 ef
**IUB-013**	808.26	1318.69 ef	510.43 ef	1.63 ef
**SLH-8**	808.26	1257.97 f	449.71 f	1.56 f
**AA-919**	808.26	1088.74 g	280.48 g	1.35 g
**IR-NIBGE-7**	808.26	976.57 h	168.32 h	1.21 h
**RH-647**	808.26	891.12 i	82.86 i	1.10 i
**HSD 0.05**	-	**79.98**	**79.98**	**0.09**

Means sharing same letter within a column are statistically non-significant (p > 0.05), HSD = honestly significant difference, BCR = benefit:cost ratio

The article "Pest susceptibility, yield and fiber traits of transgenic cotton cultivars in Multan, Pakistan" was retracted in 2022. Reasons: compromised peer review; a conflict of interest; concerns about the authorship.

## Discussion

Thirteen newly developed ‘*Bt-*cotton’ cultivars belonging to different public and private institutes of Punjab, Pakistan were evaluated for their susceptibility to sucking insects and bollworms, CLCuV attack, and seed-cotton yield and fiber quality traits under field conditions. These cultivars were included in PCCT (Punjab Coordinated Cotton Trial) for screening at different localities against insect pests, viruses and yield characteristics. Furthermore, fiber quality of these cultivars was explored. The results indicated that the maximum jassid attack was recorded for cultivar ‘FH- 647’. Similarly, the most susceptible cultivar to whitefly was ‘BS-52’. Nonetheless, the cultivars ‘AGC-999’ and ‘MNH-992’ proved the most susceptible to thrips. These results are in agreement with several earlier studies reporting differential tolerance of cultivars to various pests [28–33], which indicated significant variations in resistance levels of different cultivars of field crops like pecan, cotton, onion and mango against sucking insects. Nonetheless, recent studies have indicated that ‘*Bt-*cotton’ cultivars have been losing resistance against various insects [10–14]. Although Alam et al. [34] reported that ‘*Bt*-cotton’ cultivar ‘FH-634’ had the highest resistant to the sucking insects, we found that ‘FH-682’ was most resistant to jassid and had the highest susceptibility to whitefly. Shahid et al. [35] found that cultivar ‘FH-118’ exhibited highest resistance to thrips, whereas cultivars ‘FH-17’, ‘FH-114’ and ‘FH-179’ proved most susceptible to thrips. These results are not comparable with Singh and Lal [36] who reported that cotton varieties may respond differently to insect infestation and ‘*Bt-*cotton’ has proved resistant against highly destructive cotton pests. The differences among years can be explained by varying environmental conditions.

Regarding bollworms infestation, maximum number of spotted bollworms larvae was recorded on cultivar ‘SLAH-8’, whereas the living larvae of American bollworms were recorded on cultivars ‘RH-647’, ‘SLH-8’ and V’H-305’ in spite these are *Bt* cultivars. Although there were no rosette flowers on all of the tested cultivars from beginning to the end of crop, left over bolls of all cultivars had pink bollworm larvae. The reasons might be the low concentration of *Bt* toxin or may be due to decreased resistance in *Bt* cultivars. The results could be further confirmed on the use of *Bt* strips for the confirmation of *Bt* toxin. The results are not inconformity with that of Rao [37] who reported that *Bt* varieties provide protection against bollworms. The results in conformity with that of Babar et al. [38] who reported that ‘Bt-121’ cultivar observed spotted bollworm attack. Furthermore, these results are supported by recent studies indicating that insect resistance is slowly being lost in ‘*Bt*-cotton’ [10–14]. The results can also be compared with Bachelor and Mott [39] and Fitt [40] who reported that various lepidopteran pests couldn’t be controlled with this technology alone, although it is highly effective against *Heliothis virescens*, and *Pectinophora gossypiella* [41]. Additional chemicals have been used on a number of transgenic ‘*Bt-*cotton’ fields to control armyworm, and American bollworm [42, 43]. The results are not in comparable with that of [44–46] who reported that with the introduction of ‘*Bt*-cotton’, the farmers are getting higher yields with improved seed cotton quality due to less insect pests infestation.

The article "Pest susceptibility, yield and fiber traits of transgenic cotton cultivars in Multan, Pakistan" was retracted in 2022. Reasons: compromised peer review; a conflict of interest; concerns about the authorship.

The CLCuV incidence was recorded on cultivars ‘RH-647’, ‘IR-NIBGE-7’ and ‘VH-305’, whereas maximum yield was recorded in ‘FH-Lalazar’. A recent study indicated low yield and nitrogen use efficiency in Pakistan [16]; however, ‘FH-Lalazar’ yielded almost double of the country’s national average, indicating that it can be recommended for cultivation. Regarding fiber characteristics, maximum GOT was recorded for cultivars ‘RH-647’, whereas maximum staple length was recorded for ‘SLH-8’ and ‘IUB-013’. The fiber fineness was highest in cultivar ‘NIAB-878B’ and fiber strength in cultivars ‘BH-184’ and ‘VH-305’. Similar results for GOT [47], staple length [48], fiber strength [49] and fiber fineness [50–52] have been reported in earlier studies. The field adaptation of any new technology or cultivar depends on their economic feasibility [53]. Economic analysis indicated that ‘FH-Lalazar’ is the most promising cultivars in terms of economic returns compared with the rest of the cultivars.

## Conclusion

All cultivars were infested by different insects throughout the growing season. Finding and growing the resistant cultivar is the safest way to escape pest infestation. The study reports significant variation among tested cultivars for pest susceptibility, seed-cotton yield and fiber quality traits. However, these results are valid for Multan, Pakistan only. The cultivars could behave differently when grown in other environmental conditions. Nonetheless, current study reports that the newly developed cultivars are not complete resistant to bollworms and pest control needs to be supplemented with other control methods in the scope of IPM. Keeping in view the low pest susceptibility and high seed-cotton yield, ‘FH-Lalazar’ could be recommended for higher yield and economic returns in Multan, Pakistan. Nonetheless, regional trials should be conducted for site-specific or region-specific recommendations.
